# Language Processing Model Construction and Simulation Based on Hybrid CNN and LSTM

**DOI:** 10.1155/2021/2578422

**Published:** 2021-07-06

**Authors:** Shujing Zhang

**Affiliations:** Faculty of International Studies, Henan Normal University, Xinxiang, Henan 453000, China

## Abstract

Deep learning is the latest trend of machine learning and artificial intelligence research. As a new field with rapid development over the past decade, it has attracted more and more researchers' attention. Convolutional Neural Network (CNN) model is one of the most important classical structures in deep learning models, and its performance has been gradually improved in deep learning tasks in recent years. Convolutional neural networks have been widely used in image classification, target detection, semantic segmentation, and natural language processing because they can automatically learn the feature representation of sample data. Firstly, this paper analyzes the model structure of a typical convolutional neural network model to increase the network depth and width in order to improve its performance, analyzes the network structure that further improves the model performance by using the attention mechanism, and then summarizes and analyzes the current special model structure. In order to further improve the text language processing effect, a convolutional neural network model, Hybrid convolutional neural network (CNN), and Long Short-Term Memory (LSTM) based on the fusion of text features and language knowledge are proposed. The text features and language knowledge are integrated into the language processing model, and the accuracy of the text language processing model is improved by parameter optimization. Experimental results on data sets show that the accuracy of the proposed model reaches 93.0%, which is better than the reference model in the literature.

## 1. Introduction

Text language processing is widely used in the fields of network public opinion, crisis public relations, brand marketing, and so on. A large amount of user comment data has been accumulated on online media, which reflects netizens' emotions, attitudes, and tendencies toward hot social events, policy implementation, and products and services. Because of the strong practical value of network review data analysis, it has been deeply studied in the industry and academia. The language processing problem is studied in the data of travel blogs to help tourists choose their favorite travel destination. The classification of comment data into positive, negative, and neutral categories in language processing has become one of the key research areas in the field of natural language processing [1]. In the network environment, text expression has the characteristics of nonstandard, often using acronyms, network neologisms, spelling mistakes, grammar errors, and other problems, which brings great challenges to language processing. Methods to solve language processing problems mainly include dictionary-based methods, traditional machine learning methods, and deep learning methods [2–4].

In order to improve the accuracy of network text language processing and study the role of language knowledge and affective knowledge in the model, this paper proposes a convolutional neural network model based on the fusion of text features and language knowledge, which integrates words, parts of speech, effective dictionaries, and other external knowledge into the language processing model. Firstly, the word vector training model is used to train the word vector, and the part of speech and affective words are added to produce a variety of feature data, which is used to eliminate word ambiguity and express emotional information. Then, the convolutional neural network model was constructed, and various features were fused into the model by feature layer fusion and classification layer fusion. Finally, the neural network model is trained to evaluate the language processing effect of the model [5–9].

The neural network model has been widely used in the fields of image processing, speech recognition, and text analysis and has achieved better results than traditional machine learning methods. A classical convolutional neural network (LENETS) model is proposed and applied to image classification. In text language processing, the neural network model has also achieved very good results. The first use of convolutional neural networks for sentence segmentation class introduces deep learning into the field of text classification. LSTM cyclic neural network was used to express sentence vectors, and then discourse vectors were expressed according to sentence vectors, and discourse-level sentiment classification was carried out [10].

Since the structure of a neural network determines the effect of the model to a great extent, scholars have conducted more in-depth research on the structure of the neural network. For example, by integrating the advantages of Hybrid CNN and LSTM, attention, and other models to solve the defects of a single neural network model, Cola emotional classification neural network model is proposed. According to the characteristics of short text classification, a character-level neural network model is proposed by combining Hybrid CNN and LSTM [11].

In neural network models, word vectors are used to represent text information, and the representation ability of word vectors is an important factor affecting the model effect. Word2vec, a word vector training tool released by Google in 2013, implements two word embedding models, CBOW and SKIP DRAM, and becomes the basis for deep learning models in the field of natural language processing. According to the needs of language processing to express emotional information, the researchers improved the word vector training model. Sentiment word embedding model SSWE is used to train word vectors to improve the effect of the language processing model [12]. The word vectors containing emotional information were trained using emotion dictionaries and remote supervised information. Using word and part-of-speech concatenation, and then training vector, and disambiguation of words improve the ability of word vector text representation.

The representation and use of text emotional features play an important role in language processing. Scholars have studied a variety of emotional features and their combination methods. In this paper, a multiattention convolutional neural network model is proposed for a specific target emotion analysis task, in which three kinds of attention feature matrices are used: word, part of speech, and word position. A multichannel convolutional neural network model is proposed for the sentiment analysis task of Chinese microblogs, which integrates multiple emotion information features such as words, part of speech, and word position [13]. A convolutional neural network model combining part-of-speech information and object attentional mechanism is proposed in object-level sentiment classification.

With the research and development of deep learning theory, researchers have proposed a series of convolutional neural network models. In order to compare the quality of different models, the recognition rates of models in the literature on classification tasks were collected and sorted out, as shown in Figure 1.

Because some models do not test the recognition rate on the ImageNet dataset, the recognition rate on CIFAR-100 or MNIST dataset is given. Among them, the TOP-1 recognition rate refers to the probability that the CNN model predicts the classification with the maximum probability to be the correct category. Top-5 recognition rate refers to the probability that the CNN model predicts the correct category in the first five categories with the highest probability. Due to a series of breakthrough research results and continuous improvement according to different task requirements, the convolutional neural network has been successfully applied in different tasks such as target detection, semantic segmentation, and white language processing.

Based on the above understanding, this paper synoptically introduced the development history of convolution neural network and then analyzes the typical convolution neural network model through the stack structure, net structure of China, the structure of the residual, and attention mechanism model method, and the performance of ascension and further introduces the convolutional neural network model and the structure of the special. Finally, the typical applications of convolutional neural networks in target detection, semantic segmentation, and white language processing are discussed, and the existing problems and future development direction of the deep convolutional neural network are also discussed.

This paper proposes a joint architecture of Hybrid CNN and LSTM, which takes the local features extracted by CNN as the input of RNN to conduct sentiment analysis on short texts. In order to reduce the loss of local information and obtain the long-term dependence of the input sequence, the convolution layer and cyclic layer are used as the network model, and the short and long-time memory model is used to replace the pooling layer. The result is 6.3% better than the support vector machine method, and 1.2% better than the Hybrid CNN and LSTM with pooling layer, but sometimes the results are erratic.

In Section 2, the related work is discussed. In Section 3, a typical neural network model suitable for the analysis method in this paper is analyzed by introducing the convolutional neural network model and its operating unit. In Section 4, a language processing model based on a convolutional neural network is constructed and simulated, and the superiority of the proposed method is concluded through data analysis. In Section 5, the work of this paper is concluded, and the future work is listed.

## 2. Related Works

Choi et al. [14] proposed that the neural network model has been successful in sentiment classification, but the research on text feature representation, language knowledge representation, emotion knowledge representation, and multifeature fusion is still insufficient. Titano et al. [15] find that, on the basis of word vector representation, this paper adds external knowledge such as part-of-speech information and affective word information. Then, Rao et al. [16] clarified the convolutional neural network model structure is improved, and multiple features are fused in the feature layer and classification layer to improve language processing effects. Song et al. [17] find that word vector (WV) is trained by a word embedding model, which can represent the context and semantic information of words. Zhu et al. [18] proposed that the part-of-speech vector (POSV) was trained after combining words and parts of speech, and different vectors were used to represent different parts of speech of the same word, thus avoiding ambiguity of some words. Sentiment word vector SWV is trained with sentiment words and text sentiment tags. The research of Liu et al. [19] showed that from perceptron presentation to 2006, this stage is called shallow learning, and from 2006 to now, it is the third stage of the neural network, called deep learning. Deep learning is divided into the rapid development period (2006–2012) and the outbreak period (2012-present). In 2006, Hinton proposed the unsupervised “layer by layer initialization” strategy to reduce the difficulty of training. Moreover, a Deep Belief Network (DBN) with multiple hidden layers is proposed, which opens the curtain of deep learning.

## 3. Convolutional Neural Network Model

### 3.1. Basic Convolutional Neural Network and Operation Unit

The basic convolutional neural network includes the basic operating units of CNN: the convolutional layer, the pooling layer, the nonlinear unit, and the full connection layer. A typical CNN architecture usually alternates the convolutional layer with the pooling layer and finally outputs the results through one or more fully connected layers. In some cases, the global flat pooling layer is used to replace the full connection layer, and batch normalization and other operations are added to further optimize the performance of CNN. The structure of the convolutional neural network is shown in Figure 2:

1. Convolution Layer (CONV), also known as feature extraction layer, is mainly used for extracting features of images. It is composed of a set of convolution kernels, and the weight value of the convolution kernel can be updated according to the objective function of white motion learning. The convolutional layer is the core of the convolutional neural network
2. The pooling layer is also called the lower sampling layer. Generally, the Journal of Frontiers of Computer Skier carries out dimension reduction between two continuous convolutional layers, which can effectively reduce the number of model parameters and reduce the overfitting phenomenon of the network
3. There are maximum pooling layers and average pooling layers [20–22].
4. The nonlinear unit is composed of nonlinear activation functions, which can be divided into saturated nonlinear activation functions, such as SIGMOD function and TANK function, and unsaturated nonlinear activation functions, such as RELU function and Leaky RELU function. The nonlinear element is a nonlinear mapping of the output results of the convolutional layer, which enables the neural network to approach any nonlinear function and improves the feature expression ability of the model
5. The batch normalization (BN) is the process of transforming input data into the standard normal distribution to make the input values of nonlinear units fall into a larger value range of the gradient, so as to avoid the gradient disappearance and accelerate the convergence rate of model training
6. Fully connected (FC) layers are usually used in the classification task at the tail of the neural network, which will convert the two-dimensional vector output by the convolutional layer into a one-dimensional vector. Because the full connection layer connects all the weight of neurons in the upper layer, there are many redundant parameters that occupy a lot of hardware resources, and the spatial structure of the image is destroyed. At present, convolutional layer or Global Average Pooling (GAP) layers are commonly used to replace the full connection layer.

The application of CNN in the NLP system has achieved very good results. The convolutional layer is similar to the sliding window on the matrix, and CNN contains many complex nonlinear activation functions, such as RELU or Tank. In the classical feedforward neural network, each input of a neuron is connected to each output in the next layer, which is called the complete connection layer.

In the pooling layer, CNN extracts the image features according to the size of the convolution kernel. For example, in image classification, CNN might learn to detect edges from the original pixels in the first layer and then use the edges to detect simple shapes in the second layer, using these shapes to detect higher-level features, such as face shapes. This layer is provided to classifiers that use these advanced features. As an alternative to image pixels, the input for most NLP tasks consists of sentences and documents represented in matrix form. Each row represents a vector of one word. Usually, this vector is called the word vector. In NLP, a convolution kernel is the dimension of the word vector; that is, the width of the filter is the same as the width of the input matrix. Also, the area size may vary, but it is usually a sliding window of more than 2–5 words at a time.

The goal of RNN is to make use of the above information in text sentiment analysis by using sequence information [23, 24]. In a traditional neural network, all the inputs are independent of each other, but this approach is inefficient for many tasks in NLP [25], such as predicting the next word in a sentence. In this case, in order to predict the next word in the context, it is important to know the previous work, so the researchers came up with RNN. RNN was a great success on the NLP task. RNN has memory to capture information in arbitrarily long sequences. The network structure of RNN is shown in Figure 3.

RNN is a kind of deep neural network, which has been widely used in time series modeling. The goal behind RNN for sentence embedding is to find a dense and low-dimensional semantic representation by repeating and sequentially processing each word in a sentence and mapping it to a low-dimensional vector. It can be calculated with a simple RNN, and the output is as follows [26]:

(1) $$\begin{array}{c} o_{t}=\sum \iint_{n}n\sqrt{f\left(W_{0}h_{t}\right)}+\frac{h+w}{h\times w}, \end{array}$$

(2) ht=h+wh×w+h+1ηWhht−1+Wxxt,

where *W*_0_, *W*_*h*_, and *W*_*x*_ are parameter matrices in the neural network; *X*_*t*_ represents the input of the neural network; and *H*_*t*−1_ represents the state of the neural network at one time. Equation (2) indicates that the state at time *t* is related not only to the current input but also to the state at time *t* − 1. By analyzing the relationships between words, RNN preserves the semantics of all previous texts in a fixed-size hidden layer, while increasing the time complexity of the text. The high-level, appropriate statistics are then captured in RNN, which can be valuable for capturing the semantics of long text. RNN is a biased model where the most recent words are more meaningful than the previous words. This can be inefficient when used to capture information about the entire document. So, in order to overcome the difficulty of RNN, the Long Short-Term Memory (LSTM) model is introduced. This article uses LSTM to obtain the long-term dependency of a sentence. The LSTM network structure is shown in Figure 4.

### 3.2. Typical Convolutional Neural Network Model

In this chapter, the four network models are compared and analyzed from three aspects: model mechanism, advantages and disadvantages, and application suggestions, as shown in Table 1. It can be seen from the analysis of Table 1 that due to the different mechanisms of network models, it is necessary to select and optimize the network according to the characteristics of the network when applying the network.

#### 3.2.1. Stacking Structure Model

The stacking structure model refers to the network model formed only through the stacking of network layers without other topological structures. Early neural network models continuously improve the basic computing units of neural networks and stack them to form network models, such as Le net, Alex Net, ZF Net, VG GNet, and MSRANET. Le net forms the foundation of CNN, while the Great Normalization of Alex Net network uses RELU activation function as a nonlinear unit based on Le net and adds Dropout and Local Response Normalization (LRN) to prevent network overfitting. Due to the limitation of GPU video memory in the early stage, a stacking structure model was split and the two GPUs were used for cooperative training. With the development of a hardware platform, a single GPU platform could be used for network training without splitting the model structure anymore.

#### 3.2.2. Network-in-Network Structure Model

The Network-in-network structure model is a network model formed by using multiple branches of neural networks for operation and then connecting the results of operation of each branch. The network-in-network architecture model (NIN) was proposed in NIN and has a profound impact because it uses a small number of parameters to achieve the Alex Net effect. In the classification tasks, input features are usually highly nonlinear. NIN network induces a micro network in each convolutional layer, which can better abstract the features of each local block than stack structure. After introducing a micro network in each convolutional layer, the network depth and width are deepened and the special expression ability of the network is enhanced.

#### 3.2.3. Residual Structural Model

A residual structure model is a model structure in which a short circuit mechanism is introduced into the structure and the output of the model is expressed as a linear superposition of the input and its nonlinear transformation. In the convolutional neural network model from Alex Net layer 8, to GNet layer 19, and then to Google net layer 22, the number of layers of the model is gradually increasing, and the model performance is getting better and better, and deeper network model means better nonlinear expression ability, which can better fit complex features. Since the number of channels in the residual element is inconsistent with the output, the identity mapping cannot be used directly. However, if the 1 × 1 convolution layer is used to increase the dimension of the number of input channels, the information transmission between channels will be hindered. Dares Net adopts the residual unit structure as shown in Figure 5. In the residual path, the channel filled with zero matrices after the input feature channel is directly added to the output channel.

#### 3.2.4. Attention Mechanism Model

The attention mechanism model acquires the features that need to be paid attention to in the way of free-motion learning and inhibits the model structure of other useless features. Through the model introduced previously, it is found that a lot of work of researchers is to improve the performance of the model in the spatial dimension, while SENET can obtain the importance of each channel feature without any action, improve the weight of useful feature channels, and suppress other useless feature channels, which is a channel attention model. Combined with channel attention mechanism and spatial attention mechanism, compared with single attention mechanism model, it has better feature expression ability, and as a lightweight model, it can be seamlessly integrated into any current CNN model architecture. The attention mechanism can make the neural network have the ability to focus on its input feature subset and solve the problem of information overload.

## 4. Hybrid CNN and LSTM-Based Language Processing Model Construction and Simulation

### 4.1. Hybrid CNN and LSTM-Based Language Processing Model Construction

The framework model is composed of a convolutional neural network and recursive neural network. Firstly, the model architecture uses the word vector as the input and introduces it into the convolutional neural network to learn how to extract the high-dimensional features and then outputs it to a short- and long-time memory cyclic neural network language model and finally adds a classifier layer.  Figure 6 shows the Hybrid CNN and LSTM framework proposed in this paper:

(1) Word vector: the first layer of the network trains each word in the emotional text into a word vector with semantic information through the neural network. The input of the model is a sequence of words. In the experiment, the maximum length of the sentence is set as 100. If the sentence length is not up to the maximum, zero is used to fill it. Each emotional sentence can be represented as a 100 by 128 matrix. The matrix has semantic information and position information of words
(2) Convolution layer: in the first layer structure of the network, word vectors are used to represent each sentence as a matrix of 100 ∗ 128, which is formed by splicing simple word vectors. Convolution kernel is used to extract high-dimensional features from text. The difference between text convolution and image convolution lies in that the size of the image convolution kernel can be set arbitrarily, while the size of the convolution kernel in text convolution is twice the length of the word vector. In the experiment, the convolution kernel is set as 3 ∗ 128, 4 ∗ 128, and 5 ∗ 128, respectively. In this way, the sentence is convolved to obtain 98 ∗ 1, 97 ∗ 1, and 96 ∗ 1 sentence features, which are then spliced and filled with zeros to form a 98 ∗ 3 matrix, which is then sent into the long- and short-time memory model
(3) Cycle layer: RNN is a neural network structure specially used for sequence modeling. At each moment *t*, a loop input vector *x* and a hidden state *h* are applied, and the loop operation is
  (3) $$\begin{array}{c} h_{t}=\frac{h-w}{h\times w}+\overset{n}{\underset{t=1}{\sum }}\iint_{\sum }\sqrt[{n}]{f\left(Wx_{t}+Uh_{t-1}+b\right)}\text{d}s,\\ h_{r}=\overset{n}{\underset{t=1}{\sum }}\iint_{\sum }\sqrt[{n}]{f\left(Cw_{x}+Uh_{t-1}+b\right)}\text{d}s+\oint_{l}\left(w+h+b\right)\text{d}s. \end{array}$$
Learning the long-term dependence of an ordinary RNN is difficult because of the gradient explosion problem. LSTM overcomes this problem with input gate, forget gate, and output gate [27].
(4) Classification layer: in principle, the classification layer is a logistic regression classifier. It provides a fixed-size input from the bottom layer to fully connect to the classification layer, followed by a Softmax activation function to calculate the predicted probabilities for all classifications

### 4.2. Simulation of Language Processing Model Based on Hybrid CNN and LSTM

In the convolution neural network, there is a series of a breakthrough in the field of image classification, all applications will be different as the feature extraction of backbone network (CNN) and add a different functional unit structure to form the new application model, CNN, into to the depth of the different learning tasks, because of its excellent performance of detection effect, and gradually replace the traditional method. At present, it has become a research hotspot in the fields of target detection, semantic segmentation, white language processing, and so on.

In this paper, the language processing model is constructed. Precision, Recall, and *F*-score are used as evaluation indexes, and their calculations are shown in equations (4)–(6). Where HW is the correct number in the classification result, Hb is the number of errors in the classification result, and *F*_*n*_ is the number of incorrectly classified results in the data set of this kind of sample. *F*-score is the harmonic value of comprehensive consideration of accuracy and recall rate, reflecting the overall effect of the model:

(4) $$\begin{array}{c} \text{precision}=\oint \left(w+h+b\right)\frac{\text{HW}-\text{bW}}{\text{HW}+\text{bW}}, \end{array}$$

(5) $$\begin{array}{c} \text{recall}=\oint \left(w+h+b\right)\frac{\text{HW}}{\text{HW}+\text{bW}}, \end{array}$$

(6) F−score=h+1ηWhht−1+Wxxt+2×precistion×recallprecistion+recall.

On the basis of text features, the Hybrid CNN and LSTM model adds language knowledge such as part of speech and affective words as input data to enhance text semantic information and affective information. This experiment tests the effect of the model in sentiment classification by adjusting the number and combination of input features. WV, POSV, SWV, WV + POSV, WV + SWV, WV + POSV, and WV + POSV + SWV were obtained by combining the word vector, the part-of-speech vector, and the affective word vector.

The experimental results of feature fusion of the classification layer fusion model Hybrid CNN and LSTM are shown in Table 2.

It can be seen from Table 2 that the combination of word features, part-of-speech features, and affective word features, WV + POSV + SWV, achieves the best result of affective classification, which is significantly higher than other combinations of single features or two features. The positive category F value, negative category F value, and macro average F value of the three feature combinations reached 92.8%, 93.2%, and 93.0%, which were higher than other feature combinations, indicating that the combination of multiple features in the classification layer fusion model could improve the classification effect. The experiment proves that the accuracy of the convolutional neural network sentiment classification model can be effectively improved by adding external language knowledge such as part-of-speech features and sentiment word features on the basis of text features. The fitting curve of Hybrid CNN and LSTM is shown in Figure 7. It can be seen that the curve is relatively smooth and the gap is small in different stages, indicating that the algorithm has strong stability.

The stochastic gradient descent (CSGD) is used to train the network and the backpropagation algorithm to calculate the gradient. By adding a loop layer to the model instead of a pooling layer, you can effectively reduce the number of convolutional layers used to capture long-term dependencies. Therefore, the convolution layer and recursion layer are combined into a single model. The architectural goal is to reduce the stacking of multiple convolutional layers and pooling layers in the network to reduce the loss of detailed local information. Therefore, in the proposed model, linear units in the convolutional layer (RELU) should be used for the activation function, LSTM should be used for the recursive layer, and the hidden state dimension *d* = 128. For two datasets, the number of training cycles varies between 5 and 20. The model is compared with methods based on word embedding and convolutional architecture as well as different deep learning and traditional methods. The regularization, learning rate, and rejection rate parameters are concerned, and then, the sentence features are extracted by using the convolutional layer. The recursive layer shows the robustness of the proposed method in multiple domains. The learning rates of the convolutional layer and the cyclic layer are set as 0.01 and the loss rate is set as 0.5.

In this paper, Dropout is used as an effective method to regularize deep neural networks. The loss prevented the mutual adaptation of the hidden units constrained the 12 norms of the weight vector and inserted the Dropout module between Hybrid CNN and LSTM layer to make it more standardized.

Depth study of the classification algorithm accuracy is generally higher than that of machine learning algorithm, support vector machine in machine learning algorithms best differ with the former method by only 1.7%, and the effect of the support vector machine with Hybrid CNN and LSTM is higher than the BOW + CNN model. The reason may be the fact that a BOW + CNN model has not yet been trained to the optimal parameters, likely the fitting problem, etc. As can be seen from Figure 8, the method proposed in this paper achieves the best effect. The accuracy value of the classification algorithm is obviously higher than that of the BOW + CNN method over time, and the generated model is more stereoscopic and intuitive. Among the deep learning models, the model proposed in this paper not only has the highest accuracy but also has the lowest parameters.

In terms of feature extraction, unlike Chinese, the Uyghur language does not have natural word segmentation marks. In the Uyghur language, spaces are used as segmentation marks between words. In the experiment, Unigram and Bigram were used as feature extraction methods, respectively. From the classification results, the effect of Uyghur text sentiment classification using Bigram as feature extraction was significantly better than that using Unigram. The model proposed in this paper also achieves good results in the Uyghur language. It is 6.3% better than the support vector machine method and 1.2% better than the LSTM-CNN with a pooling layer. The validity of the proposed method is proved both theoretically and experimentally.

Although the convolutional neural network (CNN) has the advantage of learning to extract locally invariant high-dimensional features, it requires many layers of convolution to capture long-term dependencies due to the locality of convolution and pooling. This situation becomes more serious as the length of the input sequence increases. Ultimately, a very deep network with many convolutional layers is required. This article proposes a new framework to overcome this problem, in particular, to capture word information in sentences and reduce the number of parameters in the architecture. On the basis of the input word vector, this framework uses the method of combining a convolutional neural network and a cyclic neural network. Even if there is only one recursive layer, the sorting information can be retained. Therefore, using a loop layer instead of a pooling layer assumes less loss of detail in local information and more efficient capture of long-term dependencies.

The proposed method Hybrid CNN and LSTM performs well on the two datasets and achieves competitive classification accuracy while being superior to other methods. Experimental results show that the same level of classification performance can be achieved using a smaller architecture. In future research, this method is expected to be applied to other fields such as information retrieval or machine translation.

## 5. Conclusion

With the development of research on convolutional neural networks, their performance and model complexity are also improved. In this paper, a typical convolutional neural network model Hybrid CNN and LSTM with excellent performance is analyzed. The typical convolutional neural network model has made remarkable achievements and has high accuracy in image classification and recognition. It mainly includes key technologies such as increasing the width and depth of network structure and merging the attention mechanism of channel domain and spatial domain.

However, by adding some specific noises to the original image, the artificial disturbance can easily make the neural network model misclassify the image. How to solve this problem and improve the generalization ability of the model is a problem to be solved. Moreover, with the deepening of the depth and width of the neural network, the training cost gradually increases. If the prior knowledge of specific problems can be added to the model construction, the model training speed will be greatly accelerated. In addition, there is still a large space for structural research of convolutional neural networks. The improvement of model performance requires more reasonable network structure design, and the setting of super parameters of network model depends on experiment and experience, so the quantitative analysis of parameters is a problem to be solved for the convolutional neural network. Although the convolutional neural network is in a very hot stage of research, there is still a lack of complete mathematical explanation and proof about it. It is of great significance for the further development of convolutional neural networks and the solution of the defects of the current network structure to carry on the related theoretical research.

The special models listed in this paper also put forward more design ideas for the traditional convolutional neural network model:

1. Typical convolutional neural network models need lightweight design. In the past, the research of convolutional neural networks focused on algorithm design, but the specific deployment platform of its model application was not considered. The design of a hardware-friendly model structure will help to further improve the model performance, which is also the key research direction of model structure design
2. To strengthen the convolution model structure of weakly supervised or unsupervised learning, in the white realm, unsupervised learning is more common and conforms to the thinking mode of the human brain. Although unsupervised learning and weakly supervised learning have made some progress in image recognition, there is still a big gap between unsupervised learning and semisupervised learning in the accuracy of image recognition compared with supervised learning
3. To construct the multi-input convolutional neural network model structure, multi-information input can make full use of the implicit feature expression in the original data and obtain a better recognition effect with less training cost. And sharing the network structure in the recognition process can further accelerate the recognition efficiency
4. To study a more efficient feature generation method, the efficient redundant feature generation method can reduce the number of model parameters and generate more abundant feature graphs, which is also worth studying

The Hybrid CNN and LSTM model is an important research field. Typical and specific convolutional neural network models have been applied in areas such as intelligent security, virtual reality, intelligent healthcare, white driving, wearable devices, and mobile payments. The development of deep neural network models plays a key role in leading the development of science and technology and the artificial intelligence industry in the future. Future research can be carried out to further solve the existing problems and realize their application value.

## Figures and Tables

**Figure 1:** The recognition rates of models in the literature on classification tasks.

**Figure 2:** The structure of the convolutional neural network.

**Figure 3:** The network structure of RNN.

**Figure 4:** The LSTM network structure.

**Figure 5:** Dares Net adopts the residual unit structure.

**Figure 6:** The Hybrid CNN and LSTM framework proposed in this paper.

**Figure 7:** The fitting curve of Hybrid CNN and LSTM.

**Figure 8:** Comparison of display models and classification algorithm accuracy between Hybrid CNN and LSTM and BOW + CNN.

**Table 1:** Comparative analysis of four models.

Advantages and disadvantages of model mechanisms	Structures	The model's structure	Application suggestions	Stacked structure model
There is only one backbone network	Network structure is simple	Network is hard to train	Network-in-network structure model	Multiple network branches at multiple scales

It has the ability of reaggregating, except the number of parameters	It is applied to tasks with small data sets	Try to avoid applying to tight resources	The equipment is missing	Residual structural model

Is a short circuit mechanism network	It solves the problem of deep network modeling	Phenomenon of random depth	Enhance the autonomous feature extraction ability	The amount of computation

Used to build deep networks	Attention mechanism model	Channel attention and spatial attention	The performance of the original model	Generalization ability

**Table 2:** The experimental results of feature fusion of the classification layer fusion model Hybrid CNN and LSTM.

Characteristics of the combination	Negative (%)			Positive (%)			Macro average (%)		
	*P*	*R*	*F*	*P*	*R*	*F*	*P*	*R*	*F*
1	90.5	86.8	88.6	86.9	87.1	85.5	90.7	89	88.7
2	88.9	88.8	88.8	88.8	89.6	85.1	89.6	87.2	87.1
3	89.6	89.3	89.3	89.3	87.1	89.4	87.1	89.4	82.1
4	87.1	89.4	87.1	89.4	87.1	89.4	88.2	89.5	83.4
5	92.2	93.4	92.8	92.9	91.6	92.2	92.5	92.5	92.5
6	92.8	93.7	93.2	93.3	92.3	92.8	93	93	93
1.WV	2.POSV	3.SWV	4.WV + POSV		5.WV + SWV		6.WV + POSV + SWV		

## Data Availability

The data used to support the findings of this study are available from the corresponding author upon request.

## References

[1] Li X., Wang H., He H. (2019). Intelligent diagnosis with Chinese electronic medical records based on convolutional neural networks. *BMC Bioinformatics*.

[2] Liang D., Gong P., Tang X. (2019). Rapid nuclide identification algorithm based on convolutional neural network. *Annals of Nuclear Energy*.

[3] Wu P., Sun J., Chang X. (2020). Data-driven reduced order model with temporal convolutional neural network. *Computer Methods in Applied Mechanics and Engineering*.

[4] Wang H., Cao Z., Hong B. (2020). A network intrusion detection system based on convolutional neural network. *Journal of Intelligent & Fuzzy Systems*.

[5] Pak U., Kim C., Ryu U., Sok K., Pak S. (2018). A hybrid model based on convolutional neural networks and long short-term memory for ozone concentration prediction. *Air Quality, Atmosphere & Health*.

[6] Giménez M., Palanca J., Botti V. (2020). Semantic-based padding in convolutional neural networks for improving the performance in natural language processing. A case of study in sentiment analysis. *Neurocomputing*.

[7] Zhong Z., Carr T. R., Wu X., Wang G. (2019). Application of a convolutional neural network in permeability prediction: a case study in the Jacksonburg-Stringtown oil field, West Virginia, USA. *Geophysics*.

[8] Gan C., Wang L., Zhang Z. (2020). Sparse attention based separable dilated convolutional neural network for targeted sentiment analysis. *Knowledge-Based Systems*.

[9] Du C., Huang L. (2019). Sentiment analysis method based on piecewise convolutional neural network and generative adversarial network. *International Journal of Computers Communications & Control*.

[10] Bai Z., Sun G., Zang H. (2019). Identification technology of grid monitoring alarm event based on natural language processing and deep learning in China. *Energies*.

[11] Phan A. V., Nguyen M. L., Nguyen Y. L. H., Bui L. T. (2018). DGCNN: a convolutional neural network over large-scale labeled graphs. *Neural Networks*.

[12] Öztürk H., Özgür A., Schwaller P., Laino T., Ozkirimli E. (2020). Exploring chemical space using natural language processing methodologies for drug discovery. *Drug Discovery Today*.

[13] Zhai Y., Yao Y., Guan Q. (2020). Simulating urban land use change by integrating a convolutional neural network with vector-based cellular automata. *International Journal of Geographical Information Science*.

[14] Choi J., Shin K., Jung J. (2020). Convolutional neural network technology in endoscopic imaging: artificial intelligence for endoscopy. *Clinical Endoscopy*.

[15] Titano J. J., Badgeley M., Schefflein J. (2018). Automated deep-neural-network surveillance of cranial images for acute neurologic events. *Nature Medicine*.

[16] Rao X., Lin F., Chen Z., Zhao J. (2021). Distracted driving recognition method based on deep convolutional neural network. *Journal of Ambient Intelligence and Humanized Computing*.

[17] Song H., xiu-ying Han C. E., Montenegro-Marin C. E., krishnamoorthy S. (2021). Secure prediction and assessment of sports injuries using deep learning based convolutional neural network. *Journal of Ambient Intelligence and Humanized Computing*.

[18] Zhu X., Cai Z., Wu J., Cheng Y., Huang Q. (2019). Convolutional neural network based combustion mode classification for condition monitoring in the supersonic combustor. *Acta Astronautica*.

[19] Liu R., Wang F., Yang B. (2019). Multiscale kernel based residual convolutional neural network for motor fault diagnosis under nonstationary conditions. *IEEE Transactions on Industrial Informatics*.

[20] Chen M. C., Lu S. Q., Liu Q. L. (2021). Uniqueness of weak solutions to a Keller-Segel-Navier-Stokes model with a logistic source. *Applications of Mathematics*.

[21] Gao R., Yang T., Shen Y., Rong Y., Ye K., Nie J. (2020). RPI-MCNNBLSTM: BLSTM networks combining with multiple convolutional neural network models to predict RNA-protein interactions using multiple biometric features codes. *IEEE Access*.

[22] Shao J., Qian Y. (2019). Three convolutional neural network models for facial expression recognition in the wild. *Neurocomputing*.

[23] Thakur R. S., Yadav R. N., Gupta L. (2019). State‐of‐art analysis of image denoising methods using convolutional neural networks. *IET Image Processing*.

[24] Toaar M., Ergen B., Cmert Z. (2019). Waste classification using AutoEncoder network with integrated feature selection method in convolutional neural network models. *Measurement*.

[25] Gorban A. N., Mirkes E. M., Tukin I. Y. (2020). How deep should be the depth of convolutional neural networks: a backyard dog case study. *Cognitive Computation*.

[26] Ahmadi A., Tani J. (2019). A novel predictive-coding-inspired variational RNN model for online prediction and recognition. *Neural Computation*.

[27] Zhao Z., Duan H., Min G. (2019). A lighten CNN-LSTM model for speaker verification on embedded devices. *Future Generation Computer Systems*.

